# Analysis on COVID-19 Infection Spread Rate during Relief Schemes Using Graph Theory and Deep Learning

**DOI:** 10.1155/2022/8131193

**Published:** 2022-08-12

**Authors:** Ashokkumar Palanivinayagam, Ramesh Kumar Panneerselvam, P. J. Kumar, Hariharan Rajadurai, V. Maheshwari, Shaikh Muhammad Allayear

**Affiliations:** ^1^Sri Ramachandra Engineering and Technology, Sri Ramachandra Institute of Higher Education and Research, India; ^2^Department of Computer Science and Engineering, V R Siddhartha Engineering College, Vijayawada, AP, India; ^3^School of Information Technology and Engineering, Vellore Institute of Technology, Vellore, Tamil Nadu 632014, India; ^4^School of Computing Science and Engineering, VIT Bhopal University, Bhopal–Indore Highway Kothrikalan, Sehore, MP, India; ^5^Department of Multimedia and Creative Technology, Daffodil International University, Daffodil Smart City, Khagan, Ashulia, Dhaka, Bangladesh

## Abstract

The novel coronavirus 2019 (COVID-19) disease is a pandemic which affects thousands of people throughout the world. It has rapidly spread throughout India since the first case in India was reported on 30 January 2020. The official report says that totally 4, 11,773 cases are positive, 2, 28,307 recovered, and the country reported 12,948 deaths as of 21 June 2020. Vaccination is the only way to prevent the spreading of COVID-19 disease. Due to various reasons, there is vaccine hesitancy across many people. Hence, the Indian government has the solution to avoid the spread of the disease by instructing their citizens to maintain social distancing, wearing masks, avoiding crowds, and cleaning your hands. Moreover, lots of poverty cases are reported due to social distancing, and hence, both the center government and the respective state governments decide to issue relief funds to all its citizens. The government is unable to maintain social distancing during the relief schemes as the population is huge and available support staffs are less. In this paper, the proposed algorithm makes use of graph theory to schedule the timing of the relief funds so that with the available support staff, the government would able to implement its relief scheme while maintaining social distancing. Furthermore, we have used LSTM deep learning model to predict the spread rate and analyze the daily positive COVID cases.

## 1. Introduction

Novel coronavirus 2019 emerged in China in Wuhan—the capital of Hubei province in December 2019. The virus is thought to have a zoonotic origin (the spread from animal to human) as most of the initial cases are linked to Huanan Seafood Wholesale Market [1] [2]. COVID-19 is soon identified as pandemic [3]; the image at Figure 1 shows how the exponent spread of the virus at various countries over short duration of time [4]. The virus spreads from people to people who have close contact [5], the spreading is done by small droplets (which are produced by coughing and sneezing by an infected person). Infected people suffer from symptoms like fever, dry cough, and shortness of breath. Sometimes, people spread the disease without the symptoms as few of the infections may be asymptomatic. As of 10 April 2020, approximately 1.6 million cases of COVID-19 have been found positive across 209 countries, and the death from the disease is estimated at around 95,700, and the number of patients recovered is approximately 354,000 shown in Figure 2 [6]. It is also found that most of the people with COVID-19 recover fully, while the death rate is around 14.8% for ages 80+, while for other ages, it is less than 8%. Day to day, much research is done for analyzing the COVID-19 rate through various methods like the usage of EHR [7], blockchain [8], and augmented intelligence [9].

Social distancing is a nonmedical measure to prevent the spread of the coronavirus making the people stay away from each other by minimum a distance of 2 meters. The main purpose of social distancing is to avoid the number of times that people come close to each other, thus ultimately reducing the chances of an uninfected person to have contact with an infected person to break the chain and reducing the spread of this epidemic. The image in Figure 3 shows how social distancing helps to control the spread of the infection by breaking the chain. There are few artificial intelligence (AI) based study on social distancing [10].

India, despite being the second-most populous country in the world, is one of the few countries across the world which is controlling the infection as the infection rate is 1.7, which is lower than the worst affected countries [11]. On 22 March 2020, the entire nation observed Janata curfew—all the citizens were asked to stay at home and from 24 March 2020, and the entire nation went into a 21-day lockdown to prevent the spread of the infection. Figures 4 and 5 show the infection spread as of 20 June 2020 at India [12]. Early and strict lockdown made India fight against corona. It is also found that the coronavirus can stay alive outside the human body up to a maximum of 72 hours; hence, lockdown avoids people's interaction and eventually killing the coronavirus. Moreover, lockdown causes the economy of the country to be disturbed on a large scale because of lack of employee attendance. Many sectors such as micro and small scale industries, farming, and other self-employed firms needs more man power, which might cause loss of life when no proper care is taken. Lockdown is justified as a preemptive measure to avoid large losses of life. To help the citizens financially, both the center government and the respective state governments decided to give relief funds.

To avail the relief fund, the citizens should visit a few places like banks and ATMs to avail their financial support from the government. Support staff, including police and volunteers, are allotted at these places to prevent the citizens from violating the social distancing. Because of the huge population and fewer support staff, it is difficult for support staff to organize the crowd and maintain social distancing between them which is shown in Figure 6. In this research paper, the proposed algorithm makes use of graph theory to schedule the open-close timings of banks and ATMs to help the support staff to maintain social distancing between citizens. The coloring algorithm can easily visualize when the banks or ATMs should be opened or closed; the proposed coloring is based on subgraph coloring [13].

A treatment for COVID-19 is not yet found, but few researches [14] aim to find drug targeting relationships. In Feb. 2020, few health systems like UW Medicine found few drugs to cure COVID-19 [3], and these drugs need to be tested across large scale before releasing to the public. The sliding value is set as 1 to predict the daily cases; however, this is not a limitation, and the number can be increased to any positive value. The sliding value is useful in many cases; suppose if the positive case for one week needs to be found, then, the value can be set as 7.

To control the spread of the disease, the government should take measures to reduce the growth rate.  Table 1 shows the growth rate for 10 days from June 11 2020 to June 20 2020 [15].  Table 2 describes synthetic dataset. The growth rate is calculated using the formula in Equation (2). The data of daily positive cases are collected from the Indian Health Department daily circular; the future values and for the days where values are not officially released are predicted using linear regression model.

(1) $$\begin{array}{c} \text{Growth }{\text{Rate}}_{\text{dayi}}=\frac{{\text{Case}}_{\text{dayi}}‐\text{Cas}{\text{e}}_{\text{dayi}‐1}}{{\text{Case}}_{\text{dayi}}}*100. \end{array}$$

## 2. Contributions

The paper proposes a graph coloring algorithm that can schedule the open-close timings of the banks/ATMs to help the support staff to maintain social distancing between the citizens. Our contributions are as follows:

- Partition the graph representation of the country geography into subgraphs so that each subgraph represents a district
- Implement the graph coloring based on the population and the availability of support staff
- Recommend the colored graph to the government so that they can schedule the relief fund execution plan
- Predict how much reduction of COVID-19 spread rate caused by the proposed method

This paper contains six sections. Few works related to graph theory are presented in Section 2.  Section 3 contains the proposed methodology and the implementation details. We evaluate our work with some set of experiments which are discussed in Section 4.  Section 5 contains the discussion part, and finally conclusion and the future work are provided at the Section 6.

## 3. Related Works

Graph coloring is one of the active research algorithms in graph theory where a given graph G and a set of k colors [16], the objective is to color all vertices of G with any one of the colors in k, where no two adjacent vertices share the same color. The application of graph coloring is at all-disciplinary research. [17] proposes a coloring algorithm game that starts from a connected graph, and after each turn, the smallest integer k is found. The subgraph that is generated during the process is also connected. They prove that for the number of colors *k* ≥ 3, bob wins the game, and with *k* = 2, Alice wins the game. Few other researches works [18] on when Bob starts first. In other research [19], they provide proofs for dynamic coloring, in which at least one vertex of degree 2 consists of independent color. [20] proposes b-coloring algorithm in which each color has at least one vertex which is adjacent to each other. There are other research activities [21] which use the graph coloring for entropy compression methods. The graph coloring problem can be generalized to any power graph as proposed by [22].

The coloring of grid-like graphs has been investigated by [23], and they have improved the range of chromatic number usage at grid-based graphs. There are several researches in the field of network [24, 25, 26] in which they use graph coloring algorithms for increasing the efficiency of the communications. The graph coloring is done mostly in the acyclic graph, when there is a cycle; then, it requires a minimum of three colors for a cycle [27], and in most of the network-oriented applications, it is common that there is a cycle [28].

While the majority of the research is based on the acyclic graph, there are few researches on specialized graph such as edge coloring [29] and plane graph [30, 31]. One of the specialized edge coloring is rainbow coloring [32] that is when the triangular graph has three unique edge colors, and few researches provide proof for rainbow coloring [33].

## 4. The Relief Scheduling Graph Coloring Algorithm

The paper proposes a modified graph coloring algorithm in which colors are given based on the availability of support staff rather than considering neighbors alone. Before implementing the proposed model, the proposed algorithm first considers partitioning the graph representation of the country into disjoint subgraphs where each subgraph represents a district. This is because the availability of support staff can be easily measured and can be easily transported from one city to another.  Figure 7 shows how the division is made. In the figure, the vertex denotes cities, and the edge between the vertexes denotes the route between one city towards another.

Once the division is made, a dummy node has been created, and all the nodes are connected towards it in a different graph. The connection is made as per star topology [34, 35]; that is, in this new graph, all the cities are connected only with the dummy node. The edge value represents the population count of each city. The nodes in the district are the same as the number of cities in that respective area. The equation of this graph is shown in Equation (3). The procedure for constructing the star topology is shown at Algorithm 1

(2) $$\begin{array}{c} \text{Edge}\left(\text{dummy node},\text{city}\right)=\text{Population}\left(i\right). \end{array}$$

The purpose of constructing star topology is because connecting and managing the people population over cities becomes easy [36, 37]. Let the available support staff in a subgraph (entire district) be *Ns* and the total population in a city *i* is *Nci*. Let the constant value *M* denotes the maximum number of citizens that single support staff can manage at a time to maintain social distancing. The goal of the paper is to divide the existing population less than or equal to *M*, so that it becomes easy for the support team to organize the public. If the population is greater than *M*, then it will be overcrowded, and the support team cannot manage the population, and it becomes difficult to maintain social distancing. The maximum nodes in each city depends on the population and the number of nodes can be Population/(Ns∗M). For example, say *M* = 20, that is, a single support staff can manage up to 20 public citizens at a time and prevent them from avoiding social distancing. Suppose if there are 1000 support staff in a district, then they can manage up to 20,000 people and help them to maintain social distancing. So the proposed graph coloring algorithm should color the cities of not more than 20,000 populations with one color. Hence, there are two different cases arise.

### 4.1. Case 1: If Nci < *M*∗Ns

In case a single city has less population than *M*∗Ns (the maximum population that the support team can manage), then, the next city is added towards the count. The process of adding next city continues until there are no more cities left in the particular subgraph or the cumulative population reaches *M*∗Ns. If the distance of neighboring cities is more than 10 KM, then a new dummy node is created.

### 4.2. Case 2: If Nci > *M*∗Ns

For large cities, it is common that the support team cannot handle the entire population of the city, even if all the support team has involved in it. So in that case, the proposed algorithm is used to partition the city into distinct areas. The division is performed by calculating the total area of the city divided by the population. Then, either each division or combination of multiple divisions is considered based on the value of *M*. The cities in the topology are sorted based on their population in ascending order before consideration of inclusion. The Algorithm 2 shows the working model of the proposed algorithm. The Figure 5 shows the final output of the proposed algorithm. The main judgment criteria are the population of the city. If the population is less than the dummy node size, then more than one city is present in the dummy node; otherwise, one city is placed across many dummy nodes. In majority of the cases, each city is spanned across multiple dummy nodes.

## 5. Results and Discussion

In this section, we present the evaluation result of our experiment such as number of cities affected/minimum number of k (colors) required to maintain proper social distancing. We have considered the following assumptions before starting the experiment

1. The support staffs are not affected from COVID and fully vaccinated
2. The number of support staff is not changed throughout the experiment
3. There is no more than 10KM distance from each neighboring city

### 5.1. Dataset Description

In our experiment, we have used both real and synthetic datasets. In the real dataset, we consider two Indian cities. The details of real dataset are given at Table 3. Two synthetic datasets (uniform and skewed) are constructed which contains 1000 cities. The dataset description is given in Table 2. In uniform dataset, the population of the cities is randomized between 2,000 and 1, 00,000. In the skewed dataset, the population of the cities is in increasing order by a random number between 2,000 and 1, 00,000. The distribution of the population across the cities is shown in Table 4. In the experiment, only one district has been considered and as the result can be replicated to any number of districts without any restrictions. There are four different values of the number of support staff 500, 1000, 1500, and 2000 that were considered as shown in Table 3. The skewed dataset is calculated as follows: The population is randomly generated for each city, and then, the random values are sorted and assigned one by one to the cities from left to right until there are no more cities.

### 5.2. Analysis on Value of *k*

Figure 8 shows the minimum value of *k* (the colors required to color the graph) for different values of support staff and different populations. It can be noted that the required number of colors purely depends on the population, and the number of colors can be decreased when the number of support staff is increased. Since the available support staff is fixed, the government can call for additional volunteers who can help the support staffs to control the public and maintain social distancing between them.

The value of *k* denotes the number of days required to complete the relief scheme. The government goal should aim to reduce the value of *k*. As you can see in the graph coloring as per the value of *k*, the venues like ATMs and banks can remain open on specific days. That is, if two nodes are having the same color, that means that either they are present at two different districts (two separate subgraphs) or at the same subgraph. If the color is present in two different districts, that means there are two different independent support teams so they can manage to control the public parallelly at two different places. In case they are on the same subgraph, that means there is enough support team to control the public at two different places. The relief schemes should be made within the allocated short duration as it will timely help the poor, so Figure 9 shows how many support staff should be made available to complete the relief scheme. To increase the support staff, the government may call for additional volunteers.

The growth rate is the most important aspect to be considered as far as any pandemic is concerned. If the growth rate is under control, then the government is easily able to get rid of the pandemic. As discussed earlier, social distancing is the current best solution taken by all countries across the world to keep the growth rate under control. We have made a study on our proposed method and how it affects the growth rate. At few situations which include fewer support staff, then, the spread cannot be controlled. The proposed method aims to utilize the available support staff most optimally, hence maintaining social distance as much as possible.  Figure 10 shows how much the growth rate is reduced by the implementation of the proposed algorithm. Uniform dataset is used to construct the graph.

When the number of support staff and the number of additional volunteers are known, it is easy to calculate the required number of days for completing the relief schemes by the government. The formula for calculating the required number of days is given in Equation (3). Using the formula, it is found that in the two datasets, 54 and 55 days are required to complete the relief funds, respectively. Figures 3 and 7 show the number of cities which are affected without maintaining social distancing when the number of days is fixed for the uniform and skewed datasets, respectively. The data used in the experiment was *m* = 20 and Ns = 50000. When the proposed algorithm is not used, then the Ns is considered as an uniform distribution across all the cities.

### 5.3. Analysis on Spread Rate

In this subsection, we will present how the proposed graph coloring algorithm helps to reduce the spread of the coronavirus. In this analysis, we consider a few assumptions for the experiment as shown in Table 3. We assume that 25,000 is the total positive case in both the setup. As per the assumption, the relief funds should be completed within 15 days. We assume that the entire population visits the relief fund issuing location (such as ATMs and banks) once on a random day between 1 and 15. If the number of support staff is sufficient to complete the relief funds in 15 days in block, then the entire block is considered in calculating the infections. If the support staff is less, then the blocks are divided into batches, and each batch is considered at once for calculating the infections.

In the experiment, a maximum of 5,000 (in setup 1) and 10,000 (in setup 2) people can be controlled by support staff and help to maintain social distancing; since the arrival rate of the customers to the relief fund issue location is randomized, the maximum citizens saved from infection are not more than 3,284 (with the assumption parameters). The graph in Figures 11 and 12 shows how much infection is possible with and without the graph coloring algorithm. In those graphs, it can be observed that maintaining social distancing helps to reduce the infections as the proposed system helps the government to maintain the social distancing among its citizens; the graph in Figure 13 shows the how many citizens are saved from the spreading of the infection. The values present in the graph also indicate the number of citizens that were controlled by the support staff.

(3) $$\begin{array}{c} \text{Required Days}=\frac{\text{Total Population}}{M*N_{s}}. \end{array}$$

### 5.4. Analysis on Reduction of Spread Rate

The aim of this research work is to optimize the work schedule of the support staff to minimize the spread rate. In this subsection, we present the analysis of how many people can be saved from infection using the proposed method. For this purpose, we use long-short-term memory model (LSTM) [29]. The structure of LSTM is illustrated in Figure 14. LSTM is widely used in many time series prediction because of its ability to remember the past value [38] [39]. The working of LSTM is based on three gates called as forget gate, input gate, and output gate. The LSTM model is used to compute the number of affected persons based on the previous inputs. If the affected number is less than Ns∗*M*, then, the infection is saved completely, and if it is more than the Ns∗*M*, then, the difference value is considered as affected.

Forget gate decides what information should be removed from the LSTM model. It uses a sigmoid function to assign a weight between 0 and 1. A 1 represents to keep the information fully, and a 0 represents to get rid of the information completely. Equation (4) illustrates forgot gate.

(4) $$\begin{array}{c} f_{t}=\sigma \left(W_{f}.\left[h_{t-1,}x_{t}\right]+b_{f}\right). \end{array}$$

The second gate is responsible for storing new information in the LSTM model. This gate uses the weighting scheme like the forget gate along with a list of candidate values generated. The equation of input gate and the candidate generation is illustrated in the following equations:

(5) $$\begin{array}{c} \text{it}=\sigma \left(W_{i}.\left[h_{t-1},x_{t}\right]+b_{1}\right), \end{array}$$

(6) $$\begin{array}{c} C=\tan h\left(W_{c}.\left[h_{t-1},x_{t}\right]+b_{c}\right). \end{array}$$

Finally, the output gate decides the value that is going to leave the LSTM. This gate uses sigmoid for outputting the filtered information. The output value is multiplied with cell state and a tanh function as described in the following equations:

(7) $$\begin{array}{c} \text{ot}=\sigma \left(W_{0}.\left[h_{t-1},xt\right]+\text{bo}\right), \end{array}$$

(8) $$\begin{array}{c} h_{t}=o_{t}*\tan h\left(C_{t}\right). \end{array}$$

The parameters used in calculating the spread rate are the support staff count (Ns), the maximum number of people each support staff can monitor (*M*), the population of the city, and the previous 7 days of impact. We have considered the number of past values to remember as 7 (1 week). The number of hidden layers in the model is 50. We have used the Adam optimizer with batch size as 10. In the experiment, we divided the daily positive cases into two groups; first, controllable- this determines how many cases can be prevented by using the proposed graph coloring method; second, uncontrollable - this represents how many cases cannot be prevented by the proposed method. The number of past days is set to 7 because as per the WHO report, seven days is the minimum time frame for affected persons to show symptoms of COVID. The uncontrollable value is fed into the LSTM to determine the spread rate. The mean square error (MSE) is used to train the LSTM model; the equation for MSE is shown in the following equation:

(9) $$\begin{array}{c} \text{MSE}=\frac{1}{n}\overset{n}{\underset{i=1}{\sum }}{\left(y_{i}-{\ddot{y}}_{i}\right)}^{2}. \end{array}$$

where Yi denotes the actual value. This can be calculated as the number of people who are infected when the proposed graph coloring algorithm is used. Yi denotes the predicted value by the LSTM model.  Figure 15 shows LSTM model to predict the reduction of spread rate.

Figure 16 shows the prediction of LSTM and the reduction of the growth rate when the proposed graph coloring approach is used. All the data used in this experiment is shown in Table 5.

## 6. Discussion

In the corona pandemic time, it is advised to the citizens to avoid crowded places as there are more chances to get infected from the disease. Lockdowns are one of the most followed practices to avoid people gatherings and community events. However, lockdowns cause a massive economical downslide to families across the nation. Moreover, the government is taking steps to provide relief funds to the public to help them from the economic problem. There is a high chance that the social distancing will not be followed during the relief scheme operation. Hence, the government should plan the process of relief scheme properly and direct the support staff about the social distancing instructions. In this paper, we provide a graph coloring approach that helps the government to schedule the timings of the relief funds. Each color in the graph represents unique days or time, so the number of colors in the graph indicates the number of minimum days required for the government to schedule the relief scheme program shown in Figure 17. Consider a real-time example of elections where all people need to visit some common places to cast the vote. In that case, the proposed method can be useful in determining how many support staffs are need in each constituency. In this example, each constituency can be considered as one dummy node.

## 7. Conclusion

India is the second-largest populous country in the world. The available less number of support staff makes it difficult to maintain social distancing during relief schemes. In this paper, the paper has proposed a graph coloring algorithm that can help the government to open ATMs and banks according to the available support staff efficiently. The proposed algorithm has been tested on synthetic datasets by changing the values of population and availability of support staff, and the possibility of social distancing has been validated. The algorithm also recommends how many support staff are required to conduct relief schemes smoothly. In the end, the ultimate goal of maintaining social distancing is achieved. The merit of the proposed work is as follows: first, the governments can plan in advance before providing any relief scheme; second, the availability of support staff can be organized based on the need; and third, the positive cases can be controlled widely. In future work, we aim to enhance the graph coloring algorithm by migrating the excess staff to neighboring districts.

## Figures and Tables

**Figure 1:** A sample subgraph construction from three districts.

**Figure 2:** The spread of coronavirus (globally).

**Figure 3:** Number of cities affected in uniform dataset.

**Figure 4:** Coronavirus outbreak at India.

**Figure 5:** The end result of graph coloring. The image shows how the division is made using graph coloring.

**Figure 6:** The control of infection through social distancing.

**Figure 7:** Number of cities affected in skew dataset.

**Figure 8:** The minimum *k* value needed to color the graph.

**Figure 9:** The minimum number of support staff needed.

**Figure 10:** The graph shows the reduction in growth rate of covid-19 when the proposed method is implemented.

**Figure 11:** The comparison of number of infection (setup 1).

**Figure 12:** The comparison of number of infection (setup 2).

**Figure 13:** The figure visualizes the number of infections prevented from using the proposed graph coloring method.

**Figure 14:** The LSTM model used to update the COVID time series data.

**Figure 15:** LSTM model to predict the reduction of spread rate.

**Figure 16:** Growth rate comparison.

**Figure 17:** The spread of the disease. Blue dots indicate the absence of the COVID-19, and the red dots represent the presence of the disease. (a), (b), (c), and (d) denote the spread at different times when the proposed system is not used. The images at (e), (f), (g), and (h) show how the spread is controlled after the proposed system is implemented.

**Algorithm 1:** Construction of Star Topology.

**Algorithm 2:** Graph Coloring

**Table 1:** Growth rate of COVID-19 at India.

Date	+ve cases	Growth rate
June 20	411, 750	4.02
June 19	395, 838	3.87
June 18	381, 098	3.77
June 17	367, 269	3.7
June 16	354, 161	3.23
June 15	343, 075	3.01
June 14	333, 043	3.55
June 13	321, 638	3.89

**Table 2:** Synthetic dataset description.

Dataset	Number of cities	Average population
Uniform	1, 000	53, 029.45
Skewed	1, 000	52, 333.725

**Table 3:** City population details in each dataset.

Range	City count (uniform)	City count (skewed)
2000 – 5000	25	23
5001 – 10000	55	50
10001-50000	370	406
50001-70000	227	191
70001-90000	218	210
90001-100000	105	120

**Table 4:** Indian city description.

City	Number of police	Population
Greater Chennai	98, 862	8, 653, 521
Delhi	77, 965	19, 298, 507

**Table 5:** Experiment setup.

Setup	Population	*Ns*	*m*	Max # of days	Spread ratio
Setup1 Setup2	400000 400000	250 400	20 25	15 15	4.01 3.23

## Data Availability

The data used to support the findings of this study are included in the article.
